# OS-LALM-OGM Algorithm-Based Computed Tomography Image for Characteristics and Comorbidities of Patients before Transcatheter Aortic Valve Implantation

**DOI:** 10.1155/2021/3631208

**Published:** 2021-11-11

**Authors:** Wenjie Sun, Jin He, Xianzhen Tan, Yi Wang, Fei Chen, Dan Xu, An Xie

**Affiliations:** ^1^Department of Radiology, Hunan Provincial People's Hospital, First Affiliated Hospital of Hunan Normal University, Changsha 410002, Hunan, China; ^2^Department of Cardiology, Hunan Provincial People's Hospital, First Affiliated Hospital of Hunan Normal University, Changsha 410002, Hunan, China; ^3^Department of General Surgery, Hunan Provincial People's Hospital, First Affiliated Hospital of Hunan Normal University, Changsha 410002, Hunan, China; ^4^Department of Cardio-Thoracic Surgery, Hunan Provincial People's Hospital, First Affiliated Hospital of Hunan Normal University, Changsha 410002, Hunan, China

## Abstract

Based on the ordered subsets (OS), a linear augmentation Lagrangian method (OS-LALM) was constructed, which was then combined with the optimized gradient method (OGM) to construct the OS-LALM-OGM, so as to discuss application of the computed tomography (CT) images based on OS-LALM-OGM in evaluation of clinical manifestations and complications of patients before transcatheter aortic valve implantation (TAVI). The OS-LALM-OGM was compared with the filtered back projection (FBP) and OS-LALM. In addition, it was applied to evaluate the conditions of 128 patients before TAVI. It was found that the peak signal-to-noise ratio (PSNR) of OS-LALM-OGM was greater than that of the FBP and OS-LALM when the number of iterations was 5, 20, and 40, while the root mean square error (RMSD) was the opposite (*P* < 0.05). The proportion of dyspnea was the highest, 38.28%, followed by angina (19.53%) and fainting (21.09%). The long diameter of the annulus and the average inner diameter of the annulus measured by the CT image based on the OS-LALM-OGM algorithm were greatly larger than the inner diameter of the aortic annulus measured by the CT based on the FBP algorithm (*P* < 0.05); the evaluation sensitivity (95.24%) and specificity (85.85%) of CT based on the OS-LALM-OGM algorithm were obviously greater than those of X-ray, which were 84.43% and 76.77%, respectively (*P* < 0.05). In short, the OS-LALM-OGM proposed had a relatively excellent effect on CT image reconstruction. The CT image based on the OS-LALM-OGM algorithm showed a better evaluation performance for patients before TAVI than the traditional FBP algorithm, showing higher sensitivity and specificity.

## 1. Introduction

The aortic valve is a “valve” located between the left ventricle and the aorta. When the ventricles contract, the aortic valve opens and blood flows into the aorta. Aortic valve stenosis refers to the abnormality of the aortic valve structure or function caused by rheumatic fever, congenital malformations, and valve calcification, which causes restricted aortic valve opening and causes left ventricular ejection disorders [1, 2]. The disease progresses slowly, and there may be no obvious symptoms for a long time. As the disease worsens, symptoms such as angina and dizziness may appear [3]. If aortic valve stenosis cannot be treated in time, it can also lead to complications such as heart failure, arrhythmia, congestive heart failure, infective endocarditis, systemic embolism, and gastrointestinal bleeding [4]. TAVI is an interventional therapy that has emerged in recent years to treat aortic valve stenosis. It can deliver an interventional catheter through the femoral artery to deliver the artificial heart valve to the aortic valve. The area is opened to complete the implantation of the artificial valve and restore the valve function. This operation does not require thoracotomy and has the advantages of less trauma to the patient and quick recovery after surgery [5, 6]. The current clinical preoperative evaluation of TAVI patients includes clinical and aortic root anatomical indication evaluation. Imaging examinations can be used to assess the aortic root morphology and anatomical adjacency, locate the aortic valve annulus, and help doctors select patients for surgery.

CT mainly uses precisely collimated X-ray beams, gamma rays, and ultrasound together with extremely sensitive detectors to scan a certain part of the human body one by one, with fast scanning time, clear image, and other characteristics [7, 8]. The clinical use of CT will use high radiation doses to obtain high-quality images with higher resolution and better display effects, but high radiation can cause damage to the patient's body, causing cancer, gene mutations, leukemia, and other diseases [9]. Therefore, how to use the obtained noise image and incomplete projection data to reconstruct a higher-quality CT image is a hot topic for current scholars. OS is a method that uses only a subset of observation data to perform gradient calculations. Momentum terms can be introduced to speed up the convergence of the algorithm and improve system performance [10]. Gradient algorithm is a kind of momentum technology, which can solve large-scale optimization, including signal and image processing, machine learning, and communication. LALM is generally used to solve compound convex optimization, but it has the disadvantages of difficult reference selection and slow convergence [11, 12]. Therefore, the OS was adopted to optimize the LALM and then combined the OGM to construct a CT image reconstruction algorithm, so as to provide help for patient evaluation before TAVI.

In summary, CT imaging has a wide range of applications in the field of medical screening, but there are also some urgent problems to be solved. Based on this, the ordered subset (OS) was adopted to optimize the linear augmentation Lagrangian iterative algorithm into OS-LALM, which was then combined with the optimized gradient method (OGM) to construct the OS-LALM-OGM. The OS-LALM-OGM was compared with the filtered back projection (FBP) and OS-LALM and applied to evaluate the 128 patients before TAVI. The application of CT images in the evaluation of clinical manifestations and complications of patients before TAVI was comprehensively evaluated, so as to provide a good theoretical basis for imaging detection of patients before TAVI.

## 2. Materials and Methods

### 2.1. Research Objects

128 high-risk patients with severe aortic valve stenosis who were admitted to the hospital from May 2018 to March 5, 2021, were selected as the research objects, including 91 males and 59 females, aged 60–90 years old. The study had been approved by the Ethics Committee of Hospital, and the patients and their families had understood the situation of the study and signed the informed consent forms.

The inclusion criteria were defined as follows: patients with area of arterial valve less than 0.8 cm2, patients with transvalvular pressure difference of aortic valve greater than 40 mmHg, and patients with surgical contraindications.

The exclusion criteria were defined as follows: patients with incomplete clinical data, patients with psychiatric diseases, patients with transvalvular peak flow rate less than 4 m/s, and patients who withdrew from the experiment due to personal reasons.

### 2.2. CT Examination

In this study, the third-generation 192-slice force dual-source spiral CT scanner produced by Siemens (Germany) was used for retrospective ECG-gated coronary scans and large-pitch total aortic scans. The contrast agent was 370 mgI/mL iopromide. The contrast agent and saline were injected into the vein sequentially, and then the dynamic continuous same-layer monitoring scan was performed. The monitoring level was 1 cm below the tracheal bifurcation. The region of interest (ROI) was selected in the ascending aorta for CT value monitoring, and the scan was automatically triggered when the 100 HU threshold was reached. The scanning range was defined as follows: the aortic root scan covered the entire heart, and the full aortic scan extended from the entrance of the thorax to the lesser trochanter of the femur. The scanning parameters were as follows: the matrix was 512 × 512, the tube voltage was 110 kV, the tube current was 60 mAs, the CARE Dose4D automatic current was used, the layer spacing was 0.75 mm, and the layer thickness was 0.75 mm. The original images obtained were sent to the workstation for image reconstruction processing, and two senior physicians were selected for evaluation. The ALD and the annulus short diameter (ASD) of annulus were recorded, and the calculated averages of ALD and ASD can represent the AID of annulus. The diameters of the sinus and sinus tube junction, the diameter of the ascending aorta, and the height of the coronary artery opening were measured and recorded.

### 2.3. Construction of OS-LALM-OGM

Firstly, the CT image was set to the following model:

(1) $$\begin{array}{c} y=Mx+\theta . \end{array}$$

In equation (1), *y* represents the measurement data, *M* represents the forward projection operator, *x* represents the image to be reconstructed, and *θ* referrs to the noise. The penalty weighted least squares (PLWS) were incorporated to reconstruct image *x*; then, the following equation could be obtained:

(2) $$\begin{array}{c} \bar{\bar{x}}=\underset{x\geq 0}{\arg\min}\left\{\varphi \left(x\right)≜\frac{{\left\|\bar{\bar{y}}-Nx\right\|}_{P}^{2}+Q\left(x\right)}{2}\right\}. \end{array}$$

In the above equation, *N* represents the system matrix, $\bar{\bar{y}}$ represents the sine graph with noise, *P* refers to the statistical weight matrix, and *Q* means the regular term retaining the edges. Then, the edge preservation regularization function can be expressed as follows:

(3) $$\begin{array}{c} Q\left(x\right)≜\sum_{i}\lambda_{i}\sum_{n}u_{r}u_{r+e_{i}}\eta_{i}\left[{\left(B_{i}x\right)}_{r}\right]. \end{array}$$

In equation (3), *λ*_*i*_, *e*_*i*_, and *η*_*i*_ refer to the regularization parameter, the corresponding offset, and the potential function, respectively; *B*_*i*_ is the finite difference matrix in the *i*th direction, and *u*_*r*_ represents the voxel-related weight. The following equation could be obtained by converting it into a compound convex optimization:

(4) $$\begin{array}{c} \left(\bar{\bar{x}},\bar{\bar{t}}\right)\in \underset{x,t}{\arg\min}\left\{p\left(t\right)+q\left(x\right)\right\}. \end{array}$$

In the above equation, *p*() and *q*() are convex functions, *p* represents the weighted quadratic data fitting term, and *q* represents the edge retention regularization term. Then, the LALM was incorporated [13] for solution; then the following equations could be obtained:

(5) $$\begin{array}{c} x^{\left(u+1\right)}\in \underset{x}{\arg\min}\left\{q\left(x\right)+\vartheta_{u}\left(x\right)+\frac{\rho {\left\|x-x^{u}\right\|}_{R}^{2}}{2}\right\}, \end{array}$$

(6) $$\begin{array}{c} k^{\left(u+1\right)}\in \underset{x}{\arg\min}\left\{p\left(t\right)+\frac{\rho {\left\|Mx^{\left(u+1\right)}-k-d^{\left(u\right)}\right\|}_{2}^{2}}{2}\right\}, \end{array}$$

(7) $$\begin{array}{c} d^{\left(u+1\right)}=d^{\left(u\right)}-Mx^{\left(u+1\right)}+t^{\left(u+1\right)}. \end{array}$$

In equations (5)–(7), *R* represents the diagonal optimization matrix, *p*() is set as a quadratic loss function, and *ρ* represents the penalty parameter; then the previous equation could be transformed into a least squares regularization matter as follows:

(8) $$\begin{array}{c} \bar{\bar{x}}=\underset{x}{\arg\min}\left\{\varphi \left(x\right)≜\frac{\rho {\left\|y-Mx\right\|}_{2}^{2}}{2}+q\left(x\right)\right\}. \end{array}$$

If *T*(*x*)≜*p*(*Mx*) was defined as a quadratic data fitting term and can be accelerated by an OS, then the following could be obtained:

(9) $$\begin{array}{c} \Delta T\left(x\right)\approx W\Delta T_{W}\left(x\right). \end{array}$$

In equation (9), *W* represents the number of quadratic functions and Δ*T*(*x*) represents the gradient of the subset. In consideration that that the near-end mapping of the quadratic function was linear, the update of *k* can have a closed solution, which was written as follows:

(10) $$\begin{array}{c} t^{\left(u+1\right)}=\frac{\rho \left(Mx^{\left(u+1\right)}-d^{\left(u\right)}\right)+y}{\rho +1}. \end{array}$$

The following equation could be obtained by combining equations (7) and (10):

(11) $$\begin{array}{c} t^{\left(u+1\right)}+\rho d^{\left(u+1\right)}=y. \end{array}$$

Then, new equations could be found after *d* was initialized:

(12) $$\begin{array}{c} d_{\left(o\right)}=\frac{y-t_{\left(0\right)}}{\rho }, \end{array}$$

(13) $$\begin{array}{c} \bar{\bar{t}}≜t-y. \end{array}$$

In equations (12) and (13), $\bar{\bar{t}}$ represents the split residual; then the initial LALM can be obtained:

(14) $$\begin{array}{c} e^{\left(u+1\right)}=M^{\prime }\left(\rho \left(Mx^{\left(u\right)}-y\right)+\left(1-\rho \right){\bar{\bar{t}}}^{\left(u\right)}\right),\\ x^{\left(u+1\right)}\in {\text{prox}}_{\left(l/\rho \right)q}\left(x^{u}-\left(\frac{l}{\rho }\right)r^{\left(u+1\right)}\right),\\ {\bar{\bar{t}}}^{\left(u+1\right)}=\frac{\rho \left(Mx^{\left(u+1\right)}-y\right)+{\bar{\bar{t}}}^{\left(u\right)}}{\rho +1}. \end{array}$$

Then, *p*≜*M*′(*t*) was set as the split gradient; it can be optimized as follows:

(15) $$\begin{array}{c} e^{\left(u+1\right)}=\rho \Delta T\left(x^{\left(u\right)}\right)+\left(1-\rho \right)p^{\left(u\right)},\\ x^{\left(u+1\right)}\in {\text{prox}}_{\left(l/\rho \right)q}\left(x^{u}-\left(\frac{l}{\rho }\right)e^{\left(u+1\right)}\right),\\ p^{\left(u+1\right)}=\frac{\rho \Delta T\left(x^{\left(u+1\right)}\right)+p^{\left(u\right)}}{\rho +1}. \end{array}$$

The previous process was the OS-based LALM, which only needed the gradient of *T* to be updated to accelerate the ordered subset. However, there was still a problem with this algorithm; that is, the penalty parameter *ρ* value was not fixed. The deterministic downward continuation technique was applied to determine the optimal size of the parameter *ρ* value, so it could be written as follows:

(16) $$\begin{array}{c} \varpi \left(u\right)≜\left(p^{\left(u\right)}-\Delta T\left(x^{\left(u+1\right)}\right)\right)\left(\Delta T\left(x^{\left(u+1\right)}\right)-\Delta T\left(x^{\left(u\right)}\right)\right). \end{array}$$

It was assumed the iteration was restarted at the *z*^th^ iteration, and then the optimal penalty parameter *ρ* can be expressed as follows:

(17) $$\begin{array}{c} \rho_{i}=\left[\begin{array}{cc} 1, & g=0\\ \max\left[\frac{\pi }{g+1}\sqrt{1-{\left(\frac{\pi }{2g+2}\right)}^{2}},\rho_{\min}\right], & \text{otherwise} \end{array}\right]. \end{array}$$

In equation (17), *g* represents the number of iterations. This method can effectively solve the regularized least squares and simplify the selection of parameters through the deterministic downward continuation method based on the second-order damping system. However, it only used the current gradient to estimate the search direction will accumulate gradient errors, so that the reconstructed images were unstable. Based on this, the OGM was incorporated; then the CT image reconstruction can be expressed as follows:

(18) $$\begin{array}{c} \left\{\begin{array}{c} M\leftarrow E^{1/2}M\\ y\leftarrow E^{1/2}y\\ p\leftarrow Q+\kappa_{\Omega } \end{array}\right.. \end{array}$$

In equation (18), *κ*_Ω_ was the characteristic function of the convex set Ω. The above process was the constructed OS-LALM-OGM.

### 2.4. Design of Simulation Experiment

This experiment run on a real data platform. The operating environment was defined as follows: Virtual Box centos 6.6–32 bit system was installed, central processing unit (CPU) was AMD Athlon 2.99 GHz, memory was 1.75 GB, and the video resolution was 480 × 320. The (FBP) [14] and OS-LALM [15] were compared with the OS-LALM-OGM algorithm constructed. The number of OS was 40, and the PSNR and RMSD of the three algorithms under different function iteration times (5, 20, and 40) were recorded and compared:

(19) $$\begin{array}{c} \text{PSNR}=10\;\log_{10}\frac{255*255}{\left[\sum_{i=1}^{A}\sum_{j=1}^{N}{\left(x\left(i,j\right)-y\left(i,j\right)\right)}^{2}/A*C\right]}, \end{array}$$

(20) $$\begin{array}{c} \text{RMSD}=\frac{\left\|x^{v}-\overset{\leftarrow }{x}\right\|}{\sqrt{O_{\alpha }}}. \end{array}$$

In equations (19) and (20), *A∗C* represents the image size and *x*, *y,* and *A* refer to the original image, the noisy image, and the number of iterations, respectively. The larger the PSNR value meant the better the image reconstruction effect, and the smaller the RMSD value meant the better the image reconstruction effect.

### 2.5. Observation Indicators

The observation indicators included the clinical manifestations (angina, fainting, and dyspnea), complications (hypertension, diabetes, renal insufficiency, cerebrovascular disease, atrial flutter, and atrial fibrillation), CT image data, and the anatomical data of the aortic root of patients with bicuspid and tricuspid valve (ALD, ASD, AID, sinus inner diameter (SID), sinus junction inner diameter (SJID), ascending aorta inner diameter (AAID), left coronary opening height (LCOH), and the right coronary opening height (RCOH)) of the patients. In addition, the evaluation sensitivity and specificity of CTs under different algorithms were calculated, respectively.

### 2.6. Statistical Methods

The data processing was analyzed by SPSS19.0 version statistical software. The measurement data was indicated as mean ± standard deviation ($\bar{x}$ ± *s*), and the count data was displayed as percentage (%). The PSNR and RMSD of OS-LALM-OGM, FBP, and OS-LALM were compared in pairwise with single-factor analysis of variance. The difference was statistically significant at *P* < 0.05.

## 3. Results

### 3.1. Comparison on Image Reconstruction Effects of Three Algorithms

Figure 1 and 2 show the PSNR and RMSD comparisons of the three algorithms under different iteration times. The PSNR of the OS-LALM-OGM algorithm was much greater than that of the FBP and OS-LALM algorithms, and the differences was statistically obvious (*P* < 0.05), while the RMSD of the OS-LALM-OGM algorithm was smaller greatly than that of the FBP and OS-LALM algorithms, showing remarkable different in statistics (*P* < 0.05). In addition, the PSNR and RMSD of FBP and OS-LALM algorithms showed no statistical difference (*P* > 0.05).

### 3.2. Image of a Patient with Aortic Valve Stenosis

Figures 3–6 and Table 1 show the analysis of a patient with aortic valve stenosis. The diagnosis was a TYPE0 bicuspid valve, the leaflets were significantly thickened and severely calcified, the size of the French sinus was reasonable, the ascending aorta was slightly wider, the heart was horizontal, double crown height was normal, the left ventricle was small, and the myocardium was thickened, so it was determined as right femoral artery was clinically recommended as the main approach.

### 3.3. The Clinical Manifestations and Complications of Patients

Figure 7 illustrates the clinical manifestations of patients, in which 1 refers to angina, 2 refers to fainting, and 3 refers to dyspnea. It can be seen that there were 25 cases of angina in 128 patients, accounting for 19.53%, 27 cases of fainting (accounting for 21.09%), and 49 cases of dyspnea (accounting for 38.28%). Among them, the proportion of patients with dyspnea was much more than the proportions of patients with angina and fainting (*P* < 0.05).

Figure 8 illustrates the complications of patients, in which 1 indicates hypertension, 2 indicates diabetes, 3 refers to renal insufficiency, 4 refers to cerebrovascular disease, and 5 represents atrial flutter and atrial fibrillation. It revealed that 59 of 128 patients had hypertension (accounting for 46.1%), 26 had diabetes (accounting for 20.31%), 9 had renal insufficiency (accounting for 7.03%), 21 cases had cerebrovascular disease (accounting for 16.41%), and 19 cases had atrial flutter and atrial fibrillation (accounting for 14.84%). Thus, the proportion of patients with hypertension was much higher in contrast to that of patients with diabetes, renal insufficiency, cerebrovascular disease, and atrial flutter and atrial fibrillation, showing observable and meaningful differences (*P* < 0.05).

### 3.4. CT Measurement Results of the Aortic Root of the Patient

Figure 9 shows the CT measurement results of the aortic root of the patient. It discloses that among the 128 patients, 71 were bicuspid valves (accounting for 55.47%) and 57 cases were trilobular valves (accounting for 44.53%).

### 3.5. The Anatomical Data of the Aortic Roots of Bicuspid Valves and Trilobular Valves of the Patients

The anatomical data of the aortic roots of the patient's bicuspid valves and trilobular valves were shown in Figures 10 and 11. It was clear that the ALD was 29.35 ± 6.17 mm, ASD was 24.38 ± 5.82 mm, AID was 26.31 ± 4.71 mm, SID was 37.55 ± 3.86 mm, SJID was 36.24 ± 5.11 mm, AAID was 41.49 ± 4.02 mm, LCOH was 17.46 ± 3.82 mm, and RCOH was 16.37 ± 3.51 mm for patients with bicuspid valves. The ALD, ASD, AID, SID, SJID, AAID, LCOH, and RCOH of patients with trilobular valves were 28.56 ± 8.34 mm, 22.86 ± 6.41 mm, 25.29 ± 4.08 mm, 35.01 ± 4.26 mm, 32.86 ± 4.27 mm, 38.35 ± 5.21 mm, 12.85 ± 4.24 mm, and 16.02 ± 4.05 mm. The data here indicated that the patients with bicuspid valve showed no great differences in ALD, ASD, AID, SID, SJID, AAID, and RCOH (*P* > 0.05) but great difference in LCOH (*P* < 0.05) in contrast to the patients with trilobular valves.

### 3.6. Comparison on CT Image of Aortic Valve Annulus Measurement Results Based on OS-LALM-OGM Algorithm and FBP Algorithm

Figure 12 shows a comparison of CT image aortic valve annulus measurement results based on OS-LALM-OGM algorithm and FBP algorithm. It could be observed that the annulus long diameter and the average inner diameter of the annulus measured by the CT image based on the OS-LALM-OGM algorithm were significantly larger than the aortic annulus inner diameter measured by the CT based on the FBP algorithm, and the difference was statistically obvious (*P* < 0.05), while the difference between the short diameter of the valve annulus and the inner diameter of the aortic annulus measured by CT based on the OS-LALM-OGM algorithm and the inner diameter of the aortic annulus measured by CT based on the FBP algorithm was not statistically observable (*P* > 0.05).

### 3.7. Comparison on the Evaluation Performance of CT Images for Patients Based on OS-LALM-OGM Algorithm and FBP Algorithm

Figures 13 and 14 show the comparisons on the evaluation performance of CT images based on OS-LALM-OGM algorithm and FBP algorithm for patients. The sensitivity and specificity of CT evaluation based on OS-LALM-OGM algorithm were 95.24% and 85.85%, respectively, and those for CT evaluation based on FBP algorithm were 84.43% and 76.77%, respectively. Thus, the sensitivity and specificity of CT evaluation based on OS-LALM-OGM algorithm were dramatically greater than those based on FBP algorithm, and the differences were statistically great (*P* < 0.05).

## 4. Discussion

The evaluation of preoperative clinical conditions and comorbidities of TAVI has always been an important reference for clinical judgment of surgical indications. The aortic valve annulus is the key to the parameters of the aortic root. Excessive aortic diameter can cause aortic root rupture and coronary ostia, while stenosis or too small aortic diameter can cause severe valve regurgitation. As a commonly used clinical examination method, CT also plays a crucial role in the evaluation of patients before TAVI [16]. Therefore, the LALM was optimized based on OS and then combined the OGM to construct the CT image reconstruction algorithm OS-LALM-OGM, which was applied in evaluation of 128 patients with severe aortic valve stenosis. Simulation experiments found that the PSNR of the OS-LALM-OGM algorithm was much greater in contrast to that of the FBP and OS-LALM algorithms, while the RMSD was much smaller, and the differences were statistically meaningful (*P* < 0.05). Such results were similar to Østergaard et al. [17], indicating that the OS-LALM-OGM algorithm proposed had a relatively excellent effect on CT image reconstruction, so it can be used as one of the algorithms that can effectively improve the quality of CT images in the future.

Of the 128 patients, 49 had dyspnea, accounting for the highest proportion (38.28%), followed by angina (19.53%) and fainting (21.09%). This suggested that CT and ultrasound screening should be performed as soon as possible for patients with related symptoms, so as to accurately diagnose the aortic valve stenosis. Among the 128 patients, 71 cases had bicuspid valves (accounting for 55.47%) and 57 cases had tricuspid valves (accounting for 44.53%). This indicated that the proportion of severe aortic valve stenosis caused by the bivalve deformity was higher, which may be due to the difficulty of intraoperative valve release caused by calcification of the valve leaflets and uneven leaflet force in patients with bicuspid valve, and the incidence of paravalvular leakage after release was higher than that of patients with tricuspid valve [18]. The height of the left coronary opening of the bicuspid valve was greater obviously than that of the tricuspid valve (*P* < 0.05), which was different from the results of Singh et al. [19]. The reason of such difference may be that abnormal development of the left main stem may aggravate the degree of coronary artery obstruction during the operation, and the widening of the ascending aorta could lead to the occurrence of intraoperative dissection. The ALD and annulus AID of measured by CT image based on OS-LALM-OGM algorithm were significantly larger than the aortic annulus diameter measured by CT based on FBP algorithm, and the difference was statistically significant (*P* < 0.05), which may be due to the three-dimensional shape of the aortic root and the oval shape of aortic valve, and measuring the ALD and ASD separately could more closely reflect the actual inner diameter of the aortic annulus [20]. The sensitivity and specificity of CT evaluation based on the OS-LALM-OGM algorithm were significantly greater than those based on the FBP algorithm, and the differences were statistically significant (*P* < 0.05), which suggested that CT images based on the OS-LALM-OGM algorithm had better evaluation performance for patients before TAVI than CT based on the FBP.

## 5. Conclusion

Based on the OS, OS-LALM was constructed, which was then combined with the OGM to construct the OS-LALM-OGM. The OS-LALM-OGM was compared with the FBP and OS-LALM and applied to evaluate the 128 patients before TAVI. It was found that the OS-LALM-OGM algorithm proposed had a relatively excellent effect in CT image reconstruction. The CT image based on the OS-LALM-OGM algorithm showed better evaluation performance for patients before TAVI than the traditional FBP and OS-LALM algorithms, showing higher sensitivity and specificity. However, the sample size for the study was small, and there was a lack of relevant registration data for patients with severe aortic stenosis. In the future, the selection of patient samples will be increased to further explore the reconstruction effect of OS-LALM-OGM on CT images. In short, the results of this study could provide a good theoretical basis for imaging detection of patients before TAVI.

## Figures and Tables

**Figure 1:** Comparison on PSNR of three algorithms under different iteration times. ^*∗*^ indicates that the difference was remarkable in statistics in contrast to OS-LALM-OGM (*P* < 0.05).

**Figure 2:** Comparison on RMSD of three algorithms under different iteration times. ^*∗*^ indicates that the difference was remarkable in statistics in contrast to OS-LALM-OGM (*P* < 0.05).

**Figure 3:** The aortic valve and measurement results of various indicators of patients.

**Figure 4:** CT image and index measurement of patients.

**Figure 5:** The coronary artery calcification score of patients.

**Figure 6:** The angiographic position display (left coronary tangential position) of a patient.

**Figure 7:** The clinical manifestations of patients. ^*∗*^ suggests that the difference was obvious in statistics in contrast to dyspnea (*P* < 0.05).

**Figure 8:** The complications of patients (1: hypertension; 2: diabetes; 3: renal insufficiency; 4: cerebrovascular disease; 5: atrial flutter and atrial fibrillation). ^*∗*^ suggests that the difference was obvious in statistics in contrast to hypertension (*P* < 0.05).

**Figure 9:** CT measurement results of the aortic root of the patient.

**Figure 10:** Comparison on ALD, ASD, AID, and SID of patients with bicuspid valves and trilobular valves.

**Figure 11:** Comparison on SJID, AAID, LCOH, and RCOH of patients with bicuspid valves and trilobular valves. ^*∗*^ indicates that obvious difference can be found in contrast to patients with bicuspid valves (*P* < 0.05).

**Figure 12:** Comparison on CT image aortic annulus measurement results based on OS-LALM-OGM algorithm and FBP algorithm. *Note.* 1, 2, and 3 in the figure refers to the annulus long diameter, annulus short diameter, and average inner diameter of annulus measured by CT based on the OS-LALM-OGM algorithm, respectively, and 4 represents the inner diameter of the aortic annulus measured by CT based on the FBP algorithm. ^*∗*^ indicates that visible difference could be found in contrast to 4 (*P* < 0.05).

**Figure 13:** Comparison on the sensitivity of CT images to patients based on OS-LALM-OGM algorithm and FBP algorithm. ^*∗*^ indicates that the different in contrast to CT results under FBP algorithm was meaningful in statistics (*P* < 0.05).

**Figure 14:** Comparison on the specificity of CT images to patients based on OS-LALM-OGM algorithm and FBP algorithm. ^*∗*^ indicates that the different in contrast to CT results under FBP algorithm was meaningful in statistics (*P* < 0.05).

**Table 1:** The maximum, minimum, and average values of each structure of the aortic valve.

Ascending aorta Ø	Min: 39.4 mm max: 40.1 mm average: 39.7 mm
Sinotubular junction Ø	Min: 28.6 mm max: 33.6 mm average: 31.1 mm
Aortic annulus	Min Ø: 20.9 mm max Ø: 27.7 mm average Ø: 24.3 mm eccentricity: 0.24
LVOT Ø	Min: 20.2 mm max: 30.5 mm average: 25.3 mm
Sinus of valsalva height	
Aortomitral continuity length	
Annulus to apex	

## Data Availability

The data used to support the findings of this study are available from the corresponding author upon request.
